# Insights on the Dynamics and Toxicity of Nanoparticles in Environmental Matrices

**DOI:** 10.1155/2022/4348149

**Published:** 2022-07-31

**Authors:** T. Devasena, B. Iffath, R. Renjith Kumar, Natarajan Muninathan, Kuppusamy Baskaran, T. Srinivasan, Shani T. John

**Affiliations:** ^1^Centre for Nanoscience and Technology, A.C. Tech Campus, Anna University, Chennai 600025, Tamil Nadu, India; ^2^Central Research Laboratory, Meenakshi Medical College Hospital and Research Institute, Meenakshi Academy of Higher Education and Research, Kanchipuram, Tamil Nadu, India; ^3^Centre for Research and Development, Department of Microbiology, Hindustan College of Arts and Science, Chennai, Tamil Nadu, India; ^4^Department of Biology, School of Natural Science, Madawalabu University, P.O. Box 247, Oromiya Region, Bale Robe, Ethiopia

## Abstract

The manufacturing rate of nanoparticles (10–100 nm) is steadily increasing due to their extensive applications in the fabrication of nanoproducts related to pharmaceuticals, cosmetics, medical devices, paints and pigments, energy storage etc. An increase in research related to nanotechnology is also a cause for the production and disposal of nanomaterials at the lab scale. As a result, contamination of environmental matrices with nanoparticles becomes inevitable, and the understanding of the risk of nanoecotoxicology is getting larger attention. In this context, focusing on the environmental hazards is essential. Hence, this manuscript aims to review the toxic effects of nanoparticles on soil, water, aquatic, and terrestrial organisms. The effects of toxicity on vertebrates, invertebrates, and plants and the source of exposure, environmental and biological dynamics, and the adverse effects of some nanoparticles are discussed.

## 1. Introduction

There is a steady upsurge in the manufacturing rate of nanoparticles (10–100 nm) owing to their widespread applications in the fabrication of nanomaterial-based products related to pharmaceuticals, cosmetics, medical devices, paints and pigments, energy storage etc. Metallic nanoparticles were used as antibacterial agents due to their ability to induce reactive oxygen species formation and cellular damage [1]. Nanoparticles possess therapeutic applications due to enhanced permeation and retention effect [2, 3] and sensing effect due to magnetic and optical properties [4, 5]. Food industries are progressing using nanoparticles which form a barrier against gases, humidity, and other factors that could alter and reduce food stability [6]. Iron oxide NPs are used in biofortification, while Cu(OH)_2_ nanoparticles are used as an eco-friendly pesticide in the field of agriculture [7, 8]. Nowadays, nanoparticles have been used to a greater extent in sunscreen and sports equipment due to their unique properties [9, 10]. Apart from the abovementioned applications, nanoparticles are used in bone reconstruction [11], car tire reinforcements, speakers' heat transfer [12], etc. The production rate of different types of nanoparticles is in the following order: titanium oxide and silicon dioxide nanoparticles > cerium oxide nanoparticles > zinc oxide nanoparticles > carbon nanotubes >silver nanoparticles [13–15]. An increase in the production rate of nanoparticles enhances their release of nanoparticles in our environment (Figure 1). As a result, the following aspects have become the important factors of nanotoxicology [16]:

1. The potential source of exposure.
2. Various analytical methods to quantify the environmental concentrations.
3. The fate of nanoparticles in the environment (aquatic and terrestrial living beings).
4. Adverse effects of nanoparticles on biological systems such as bioaccumulation and toxicity.
5. Possible nanotechnological strategies to combat nanotoxicity.

The environmental effects of nanoparticles are mainly attributed to their small size, high surface area, high surface reactivity, high aspect ratio, and diverse morphology. Studies reveal that partially functionalised metal-based nanoparticles and carbon-based nanoparticles are present in the environment [17–19]. Topics such as nanometrology, dosimetry, transformations, persistence, and bioaccumulation of nanomaterials in the complex environmental media have become very important facets of environmental nanotoxicology studies for the current industrial era [20–22]. Hence, our review systematically focuses on the source of exposure, environmental and biological dynamics, and the adverse effects of nanoparticles, whose production rate is constantly in the hike.

## 2. Sources of Nanoparticles Contributing to Environmental Toxicity

The environment of the living system such as plants, aquatic organisms, and terrestrial organisms including humans are exposed to nanoparticle candidates primarily via three sources [23–25], namely production source [26], application sites, and disposal sites [27]. The emission pathway and the release pattern usually vary for every type of nanoparticles. Titanium dioxide (TiO_2_), zinc oxide (ZnO), and silver (Ag) nanoparticles are regarded as the major OECD (Organization for Economic Co-operation and Development) priority materials. Hence, nanotoxicologists and ecotoxicologists are currently focusing on the toxicological properties of these specific OECD relevant materials. TiO_2_ and ZnO nanoparticles are major constituents of cosmetics that are ultimately released into the water. These nanoparticles are mainly released into the environment during water treatment process and hence they mainly accumulate in the soil [28, 29]. TiO_2_ nanoparticles are reported to induce size-dependent toxicity to algal species. ZnO and silver nanoparticles were however reported to undergo ready dissolution and their ions were found to be toxic to the aquatic organisms [30].

Aluminium oxide/alumina (Al_2_O_3_) nanoparticles are among the most abundantly produced chemical in nanosized particles, estimated to account for approximately 20% of the world market of nanoparticles. Alumina nanoparticles' production rises due to their application in catalysis, structural ceramics for reinforcements, polymer modification, functionalisation of textiles, heat transfer fluids, and wastewater treatment. In addition, Al_2_O_3_ nanoparticles have shown wide biological applications in biosensors, biofiltration, drug delivery, and antigen delivery for immunisation purposes. There is evidence that exposure to aluminium may also contribute to an increase in oxidative stress, inflammatory events, and/or the breakdown of the blood-brain barrier (BBB). Al_2_O_3_ nanoparticles prepared by using micro-emulsion methods and conventional sintering processes were reported to decrease the viability of various cell lines (VERO, HEP 2, A549, and MDA MB 231). Further, the aluminium oxide nanoparticles induced bacterial cell death. The attachment of alumina nanoparticles to the surface of the cell membrane and subsequent disturbance in cellular permeability and respiration were proposed mechanism of action [31].

Carbon nanotubes (CNTs) are widely used in the aerospace, automotive, and electronics industries because of their stability and enhanced metallic and electrical properties. CNTs are also being investigated for biomedical applications such as drug delivery systems and biosensors. CNTs are well known for oxidative stress, inflammation, apoptosis, pulmonary inflammation, fibrosis, and granuloma in the lungs. So, it is essential to consider the chronic toxicity of CNTs before using them for various biomedical applications. The toxicity of CNTs has already been reviewed [32]. Time-dependent pulmonary toxicity due to inhalation of multi-walled carbon nanotubes (MWCNTs) was evaluated by the bronchoalveolar lavage fluid (BALF) and histopathological analysis. MWCNTs increased cell count, neutrophils, lymphocytes, lactate dehydrogenase, alkaline phosphatase, protein, and cytokines (tumor necrosis factor-alpha (TNF-alpha) and interleukin 4 (IL-4)) with a contaminant decrease in the cell viability and alveolar macrophage count BALF on days 1, 7, and 14 postexposure, when compared to control rats. Histopathological analysis revealed inflammation, fibrosis, and granuloma in the lungs of MWCNT-treated rats on days 7 and 14 postexposure. Thus, it could be inferred that MWCNT induces inflammation, fibrosis, and granuloma characterised by the progressive elevation of TNF-alpha and IL-4. MWCNT accumulates in the lungs and tracheobronchial lymph nodes (TBLN) [33].

Coal is the main fuel source widely used in power plants for electricity generation, due to its abundance and low cost. Combustion of coal produces coal fly ashes (CFAs) containing toxic constituents such as metals, polycyclic aromatic hydrocarbons, and silica. The worldwide annual production of CFA is estimated at around 300–350 million tonnes through the combustion of 3,000 million tonnes of coal [34]. As revealed by characterisation techniques such as EDAX, atomic force microscopy (AFM), X-ray diffraction, and scanning electron microscopy, CFA consists of nanoparticles of around 50 nm, so-called CFA-Nps. CFA-Nps inhibit cellular metabolism in a dose-dependent manner at concentrations varying from 13 to 800 micrograms per ml. After 48-h exposure, the Hep2, A549, and HepG2 cell lines were found to be more sensitive to CFA-NPs at varying levels. The IC_50_ value of CFA-NP-treated Hep2, A549, and HepG2 cells was found to be 397, 243, and 259 micrograms per ml, respectively [35].

The rapid increase in motor vehicle usage is contributing to high levels of urban air pollution which constitute the main source of fine and ultrafine particles, having a serious impact on our urban air quality and public health. The toxicity of vehicle exhaust nanoparticles was reviewed in which diesel exhaust nanoparticles (DENPs) and petrol exhaust nanoparticles (PENPs) were identified and characterised in vehicle exhaust samples by Durga et al. [36]. These samples were reported to be toxic to monolayer culture of various cell lines (HT29, VER, HEP2, A459, and MDA MB23) as indicated by a decrease in cell viability [37]. In vitro exposure to PENPs induced significant oxidative stress, together with membrane leakage, lipid peroxidation, cell inflammation, and protein release, all of which may be the reason for cellular toxicity. Thus, it could be stated that PENPs have the potential to induce toxicity via oxidative stress and inflammation [38].

## 3. Tools for Analysing Nanoparticles in the Environment

Improved nanometrology is imperative for understanding the environmental concentrations of nanomaterials and for allowing accurate dosimetry in ecotoxicology testing. Suitable metrology for imaging and measuring the accurate concentrations of nanoparticles of environmental relevance is needed to assess the exact toxicological effects in the biological systems of both vertebrates and invertebrates [39]. This would help analysing the dose-response relationship more exactly. Even the currently available techniques have various limitations such as poor sensitivity, deprived resolution, and absence of completely quantitative data when using complex environmental samples. Still, surface characterisation and determining concentration of nanoparticles are essential to understand the fate of nanoparticles in the environment and food chain [40]. So far, there is no direct analytical technique to quantify the concentrations of nanoparticles in the environment. However, measurements can be done with the aid of computational modelling methods [29, 41]. There is also a need to differentiate manufactured nanoparticles from the particles already present in the tissue of the organisms considered for ecotoxicity studies. This is challenging; however, isotopically labelled nanoparticles and mass spectroscopy-based approaches are crucial in analysis and in yielding relevant data [42].

Probabilistic approaches are of greater significance [43]. This method involves the time-dependent flow of specific nanoparticles in technical modules and environmental compartments enabling the measurement of several nanograms to micrograms of nanoparticles in water samples. This method deals with the dynamic input rates, in-use stocks, and the continuous rise in production volumes [44]. This method is highly suitable for titanium oxide and zinc oxide nanoparticles.

Single-particle inductively coupled plasma mass spectrometry (sp-ICP-MS) is an analytical technique used for the quantification of certain nanoparticles in the environment. Inorganic engineered nanoparticles such as metal nanoparticles including gold, silver, and copper can be quantified by sp-ICP-MS [45]. Surface active nanomaterials in soil samples containing more than one element such as core-shell nanocomposites can be analysed using a multi-element technique, for example, sp-ICP-Time of Flight (ToF)-MS [46, 47].

Sizing and quantification of nanoparticles in the environmental media are also possible by using hydrodynamic chromatography coupled with UV-visible, fluorescence, and inductively coupled plasma mass spectrometry detectors [47, 48]. Nanoparticles tracking analysis and hyphenated methods such as field flow fractionation with inductively coupled plasma mass spectrometry (FFF-ICP-MS) and single-particle inductively coupled plasma mass spectrometry (SP-ICP-MS) are analytical tools of the modern era that are highly relevant to nanoecotoxicology studies [49, 50]. Nanoparticle tracking analysis is capable of providing more accurate data than the dynamic light scattering. SP-ICP-MS enables the single and ensemble analysis of particle number and concentration on an ion-specific basis. This technique is in fact used for the analysis of nanomaterials accumulated within biological cells [51, 52].

Electron microscopy imaging of tissue slices is very labour-intensive. However, fluorescent polystyrene microspheres can be used as probes for tracking the cellular uptake of nanoparticles in the juvenile stages of fish. SC-ICP-MS is used for the direct particle detection in alkali-digested tissue samples of environmental relevance [52, 53].

Targeted Raman spectroscopy has been able to recognise intact metal oxide nanoparticles such as ceria, zinc oxide, and titania in or on the surface of fish gills from waterborne exposures. This is highly useful for studying the bioavailability of nanoparticles in fish gills.[54]. Techniques such as gamma spectrometry (pulse-chase experiments) and autoradiography are useful in investigating the trophic transfer of nanomaterials in addition to uptake and assimilation studies. For example, the uptake, assimilation, and trophic transfer of dietary nano-CeO_2_ particles (containing gamma-emitting radioisotope Cerium-141) along a freshwater food chain represented by an alga (*Pseudokirchneriella subcapitata*), a grazing snail (*Potamopyrgus antipodarum*), and a prawn (*Macrobrachium australiense*) were studied by Cresswell et al. [55]. The study however substantiated the rapid elimination of nanoparticles in snail and the prawn suggesting the absence of assimilation in these organisms. Micro-X-ray fluorescence spectrometry has the ability to reveal the presence of metal nanoparticles in the freshwater organisms. Such studies on freshwater Asian clam *Corbicula fluminea* reveals the presence of gold nanoparticles in the gut epithelium [56].

Electron microscopy (SEM and TEM) can be used as a complementary technique for elucidating size and structural information of environmental nanoparticles [57]. TEM is useful for getting a clear image of electron-dense particles such as metallic nanoparticles. TEM images are used to obtain idea on the endocytosis pathway of cellular uptake of silver nanoparticles in aquatic organisms which feed on sediment deposits rich in silver nanoparticles. TEM images and EDAX data can reveal clear electron-dense zones of silver nanoparticles in the apical plasma membrane, endocytic pits, and in endosomes of the *Nereis diversicolor* [58]. Transmission electron microscopy is used for imaging nanoparticles such as carbon nanotubes and copper oxide nanoparticles inside the gut. Zhu et al. and Heinlaan et al. have imaged the nanoparticles in *Daphnia magna.* Single-walled carbon nanotubes and copper oxide nanoparticles were reported to accumulate in the gut lumen and midgut [59, 60].

Coupling electron microscopy with other techniques are also useful in the analysis of environmental nanoparticles in tissue samples. For example, energy-dispersive X-ray spectroscopy (EDAX) and electron energy loss spectroscopy (EELS) are used for the quantification and speciation of nanoparticles in tissue samples [61, 62]. However, even at relatively high concentrations of nanoparticles, the probability of single nanoparticle imaging in an electron micrograph of a cell such as the gill cell of a fish is undoubtedly a challenging task due to possibility of false negative results.

Isotope labelling techniques are useful for determining the bioavailability, bioaccumulation, and their relation to toxicity of nanoparticles. Croteau et al. have reported the importance of isotope labelling strategies for the determination of bioaccumulation and toxicity of copper oxide nanoparticles in freshwater invertebrates following waterborne and foodborne exposure. It was concluded that diet-borne copper oxide nanoparticles are more deleterious readily than waterborne particles [63]. Tools that are available to characterise nanomaterials in environmental samples are shown in Table 1.

Modelling nanoparticles in the environment was commenced by [64], who presented the first quantitative approach for assessing nanoparticle release and concentrations for environmental media. He described the theoretical basis on the nanoparticle release quantification that opened the field for several subsequent modelling studies. Several algorithms were developed for calculating the predicted environmental concentrations for a series of nanoparticles in water, biosolids, and soils. Due to a virtually complete lack of empirical information on nanoparticle production and use amounts, the calculations were fully based on a hypothetical model input and therefore not further used in evaluation. Mueller and Nowack [29] for the first time used a material flow analysis (MFA) to replace hypothetical calculations. Park et al. [65] employed emission and atmospheric dispersion models for their work on nanosized CeO_2_ emissions from its use as a diesel additive. Blaser et al. [66] presented modelled concentrations of Ag originating from the use of biocidal Ag applications including nano-Ag. Koelmans et al. [67] made the first steps in environmental fate modelling for carbon-based nanomaterials in sediments by combining the output of Mueller and Nowack's release model with mass balance calculations involving agglomeration, sedimentation, and burial nanomaterial in the deeper layers of the sediment for the first time. Gottschalk et al. [68] used a probabilistic material flow analysis (PMFA) approach [69] built on Monte Carlo (MC) computer simulations for assessing predicted environmental concentrations of five nanomaterials (TiO_2_, ZnO, Ag, CNT, and fullerenes) in water, sediments, biosolids, soils, and air. Musee [70] used a deterministic and scenario-based MFA to calculate nanomaterial emissions from cosmetic products into the water and terrestrial environments. Johnson et al. [71] estimated the predicted environmental concentrations of sunscreen TiO_2_ for soils by basing their PEC modelling on their own measured concentrations in biosolids. Arvidsson et al. [72] proposed a particle flow analysis approach (PFA) to assess anthropogenic nanomaterial release into the environment.

## 4. Environmental Dynamics of Nanoparticles

The rapid increase in the environmental concentration of nanoparticles, high bioavailability [73], and novel behaviour of nanoscale materials in the environment and ecosystem are responsible for the deleterious biological effects of nanoparticles [24, 74, 75]. In addition, a rapid hike in the production rate of nanoparticles is estimated to rise further thereby increasing their eventual toxicity in the environment [76]. Physiochemical properties of nanomaterials such as size, shape, specific surface area, elemental composition, surface functionalisation, and crystalline structure are also the major determinants of their environmental dynamics which leads to eco-nanotoxicity and bio-nanotoxicity [77, 78]. Once the nanomaterials are released into the environment, their tendency to aggregate, surface binding ability, potential to release toxic metal ions, capacity to passivate, or capability to interact with various environmental or biological constituents such as humic substances, (muco)polysaccharides, and cellular debris will change. As a result, their bioavailability and toxicity will also change [79–81].

Once the nanoparticles enter into the environment, they undergo dynamic transformation. Apart from the properties of nanoparticles, the environmental parameters such as pH, ionic strength, organic and inorganic colloids, temperature, etc., can also regulate the transformation process [82]. Three major transformation processes, namely physical, chemical, and biological transformations, can clearly explain the fate of nanoparticles in the environment [83].

1. Physical transformation includes aggregation, agglomeration, sedimentation, and deposition (in porous media).
2. Chemical transformation includes dissolution and subsequent speciation changes, redox reactions (oxidation and sulfidation), photochemical reactions, and corona formation.
3. Biological transformations that encompass biodegradation and biomodification.

Various factors such as the pH, the ionic strength, the presence of divalent ions, the type/concentration of organic matter, and the quantity of the engineered nanoparticles strongly influence the aggregation process [84–86]. However, the presence of natural organic matters such as humic acid and fulvic acid are known to block aggregation [87]. Homoaggregation was reported to be insignificant at realistic environmental concentrations (<1 *μ*g/L) and relevant timescales, while the heteroaggregation was quantitatively significant due to the higher concentrations of natural colloids in the environmental media. Natural organic matter is capable of replacing the surface coating of the nanoparticles and subsequently causing electrosteric repulsion and stability [88]. Merrifield et al. have also reported that the aggregation kinetics are strongly related to the initial concentration (in particular the number concentration) of the dispersed nanoparticles [89]. Measurement of the number concentration of nanoparticles and the nanoparticle mass (size) using SP-ICP-MS clearly reveals that the aggregation and the dissolution of nanoparticles depend on the concentration and the mass [62]. It was also reported that the aggregation of nanoparticles can increase the accessibility of the particles to the biomass or the ingestion rate, both of which raise the bioaccumulation [63, 90]. In marine water, nanoparticles are sterically stabilised. This leads to polymer entanglement and bridging thereby promoting aggregation [91, 92]. In the ecotoxicology community, adsorption phenomena involving the binding of metal on fish gills is influenced by physical factors such as the net charge of the surface, ionic mobility of the counterions in the surrounding medium (which in turn is partly defined by charge density and the hydrated ionic radius of the ion), and competition with other ions in the medium such as H^+^ [93]. Thus, it could be understood that the surface charge of the nanomaterials alters their ecotoxicity.

Quik et al. have demonstrated that the natural organic matters (colloids) are responsible for the sedimentation of nanoparticles in freshwater samples [94]. Quik et al. have also assessed the exposure of aquatic organisms to engineered nanoparticles and reported first-order kinetics for both sedimentation and dissolution [95].

Dissolution refers to the release of specific ions from the parent nanomaterials which in turn cause deleterious effects to the cells. Bacteriolysis is an important example of dissolution-based effect. Silver nanomaterials are iconic in releasing ions for killing bacteria which is responsible for the well-known antibacterial activity of silver nanomaterials. However, other factors such as surface functionalisation, shape, and size of the nanoparticles determine the transport, bioavailability, and the rate and extent of dissolution [96]. The following factors influence the solubility and dissolution of the nanoparticles, which in turn has an effect on their fate and toxicity in the environment: chemical nature of the nanoparticles [97, 98], size of the particles [99], surface coating [100], doping [101], and presence of natural organic matter [89, 102]

Solubility and dissolution are very low for carbon-based nanomaterials and inorganic nanomaterials. Hence, solubility does not contribute to their toxicity. However, for metal nanoparticles such as silver, copper oxide, and quantum dot exert their adverse effects due to their direct biological interaction and their accumulation within the cells. Their toxic effects are determined by the intermediate dissolution and solubility of their ions and particles as well [103]. Solubility contributes to toxicity for zin oxide nanoparticles. For carbon-based NMs and many inorganic NMs such as ceria and titania, whose solubility is low, dissolution and solubility become less important.

Sulfidation is a method of chemical transformation that involves surface modification by sulphide group that is available in wastewater treatment effluent and sediments. This process is an oxygen-dependent reaction, more predominant among metal nanoparticles which can alter the particle size, surface charge, and solubility and morphology [104]. Subsequently, the fate and the bioavailability of the metal nanoparticles get altered. [105, 106] For example, sulfidation of silver nanoparticles to silver sulphide reduces the toxicity [107]. Sulfidation of zinc oxide nanoparticles enhances the aggregation by reducing the surface charge [108]. Copper oxide (CuO) nanoparticles undergoes slow sulfidation reaction forming CuS that releases more quantity of copper ions as compared to the precursor nanoparticles resulting in more toxicity to aquatic biota [109, 110]. Silver, iron oxide, and ceria nanoparticles are prone to redox transformations. Photochemical oxidation of nanoparticles was reported to play a role in the bacterial toxicity and hence exploited as an important antibacterial mechanism [111, 112]. Nanoparticles such as carbon nanotubes, fullerene, TiO_2_, and ZnO are photoactive which get excited by light and generate reactive oxygen species (superoxide anions, hydroxyl radicals, etc) that are hazardous and toxic to the living organisms [82]. Dissolution, homoaggregation, heteroaggregation, fragmentation, sedimentation size exclusion, straining, deposition, and convective transport are the factors governing the fate of nanoparticles in soil [113]. In the native environment, redox reaction comprises of oxidation-reduction reactions. The coupled process of oxidation and reduction reaction involves the transfer of electrons between the reacting chemical components and this is influenced by environmental conditions such as pH and existence of electron donors (reducing agent) or acceptor (oxidising agent) [114].

Over the last era, many reports have explored the transport of nanomaterials through soil using natural soils, and columns containing inert stationary phases such as quartz beads in columns and appreciated the fate of nanoparticles in terrestrial system [114]. For example, single-walled carbon nanotube through porous media was explored by Jaisi et al. [115]. Fang et al. determined the fate of titania nanoparticles in saturated homogenous soil [116]. Zinc oxide nanoparticles showed higher rate of dissolution [117]. Dissolved zinc oxide nanoparticles transform into a mixture of species such as ZnS, Zn_3_(PO_4_)_2_, Zn-cysteine, Zn-substituted ferrihydrate, and Zn^2+^ adsorbed to mineral surfaces [118, 119]. Carbon-based nanoparticles (carbon nanotubes, fullerene, and graphene) generally do not undergo hydrolysis instead they dissolve via photolysis or microbial decomposition [120, 121]. High concentrations of colloids suspended in the soil pore water enables greater heteroaggregation of nanomaterials in soil, while homoaggregation is comparatively lesser. Consequently, the straining will be increased and diffusion will be increased. However, both the mode of aggregations can be inhibited by natural organic matter in soil porewater [122]. This concept was reported by studies using ceria nanoparticles [123], engineered silver nanoparticles, gold nanoparticles [124, 125], carbon nanotubes, hematite nanoparticles [126], and titanium dioxide nanoparticles [127].

Carbon-based nanomaterials such as carbon nanotubes get retained in the soil and cause significant straining [128, 129]. Fullerenes interact strongly with organic matter in the soil and get retained [130, 131].

Biodegradation of nanoparticles are more familiar in carbon-based nanomaterials such as graphene oxide, CNTs, and fullerene derivatives. Graphene oxide sheets are susceptible to degradation by neutrophil, myeloperoxidase-induced degradation producing noncytotoxic and non-genotoxic product [132]. Pristine single-walled carbon nanotubes undergo layer-by layer degradation in the presence of fungal manganese peroxidase and generate carbon dioxide [133]. Similarly, multi-walled carbon nanotubes are also susceptible to horse radish peroxidase-mediated degradation [134]. Basidiomycete fungal enzymes degrade C60 fullerol particles and decompose them [135].

Next to biodegradation, biomodification plays a role in determining the fate of environmental nanoparticles. During biomodification, the natural bioorganic molecules in the environment adsorb to the surface of the nanoparticles forming a new moiety called eco-corona. The sources of these biomolecules in the environment are microbes, plants (phytoplanktons), and animals (zooplanktons) [136]. Biomolecules of corona are made of polysaccharides, proteins, lipids, nucleic acids, etc [137]. Eco-corona may be hard or soft. Hard corona (strong corona) are directly and strongly bound to the nanoparticles, while soft corona (weak corona) is away from the nanoparticle core and bound to the hard core [138]. Eco-corona is a dynamic entity capable of exchanging its constituent biomolecules with the surrounding environmental matrices [139]. Eco-corona is capable of reducing the generation of reactive oxygen species during the interaction of nanoparticles with the zooplankton or the phytoplankton [140] or capable of altering the aggregation and dissolution behaviour of nanoparticles [141, 142]. In the context of toxicity, eco-corona is capable of minimising the toxicity of nanoparticles in various organisms such as algae, plants, and zebra fish [143–145]. As far as the water matrix is concerned, nanomaterials are highly available to the aquatic organisms at >10 m depth than at the surface [146].

## 5. Biological Fate of Nanoparticles

As mentioned earlier, the nanoparticles undergo dynamic transformation in different environmental matrices. Hence, the living systems in the environment are more susceptible to the effects of transformed nanoparticles (Table 2) rather than the pristine counterparts. Nanomaterials easily influence the aquatic and the terrestrial health probably due to their novel behaviour contributed by:

1. high surface reactivity;
2. spatial constraint of electronic properties;
3. high specific surface area;
4. easy transport mechanism in the media;
5. effective formation of interface with subcellular organelles of the living cells.

For example, nanoparticles that are tightly constraint in size and oxidation state are capable of giving different algal transcriptomic and metabolomics responses when compared to bulk counterparts [75].

Dynamic interaction of environmental nanoparticles with the biomolecules of the biological organisms results in a new entity called “bio-corona” which is analogous to eco-corona in the environment [137, 147]. The comprehensive details about bio-corona and nano-bio-interfaces are beyond the scope of this review and already discussed elsewhere [148–150]. Biodegradation, macromolecule-mediated formation of nanoparticles, and bio-corona/nano-bio interactions are the principal biological mediated transformations in the environment. The rate and relative significance of these processes depend on the interaction of nanoparticles with extracellular enzymes, extracellular polymeric substances, and microbes. The fate, transport, and potential ecological risks associated with the nanoparticles released into the terrestrial and aquatic ecosystem is determined by the biodegradability of polymer coating material, the type of underlying core/particle and the dominance/population of a particular microbial community [151]. Nevertheless, detailed studies are inadequate about the biodegradation potential of microbes for various organic polymer coatings present on different nanoparticles and subsequent transformation of nanoparticles under environmentally relevant conditions.

### 5.1. Aquatic Ecosystem-Invertebrates

Increased usage of engineered nanoparticles (ENPs) in industrial and commercial applications will inevitably end up in the mixing of these nanoparticles' aquatic environment. Based on a literature review and an overview of toxic effects of ENPs in aquatic system, it could be inferred that invertebrates are sensitive and relevant organisms for assessing the nanoecotoxicological effects of nanoparticles. Experiments conducted using invertebrate model helps one to advance the knowledge on bioavailability, bioaccumulation, and toxicity [152].

Invertebrates show bioaccumulation of nanoparticles. For instance, silver nanoparticles were internalised into the gut epithelial cells of estuarine polychaete *Nereis diversicolor*. In *Daphnia magna* and *Lumbriculus variegatus*, Khan et al. have investigated the accumulation dynamics and acute toxicity of silver nanoparticles. Silver nanoparticles were reported to enter into the cells via endocytosis and accumulate as inorganic granules, organelles, heat denatured proteins, and metallothionein fraction. Metal modelling approaches like biotic ligand model (BLM) and tissue residue approach (TRA) can be used to establish the link between uptake, accumulation, and toxicity of nanoparticles. Khan et al. have studied the bioaccumulation dynamics of silver nanoparticles functionalised with PVP, PEG, and citrate in comparison to dissolved Ag, in *Daphnia magna* and *Lumbriculus variegatus* [58, 153].

Bioaccumulation in invertebrates depends on various material properties such as the composition, size, and solubility and the environmental dynamics (dissolution, aggregation) of the nanomaterials. Nanoparticles of gold, titania, and silica are less bioavailable and less toxic in invertebrates. Nanoparticles of copper oxide, zinc oxide, and silver possess high bioavailability and high toxicity [83]. Lesser the particle size greater the bioaccumulation, probably due to greater bioavailability [154].

Next factor that determines bioaccumulation in invertebrates is the solubility. For example, silver in dissolved form is more bioavailable and showed higher bioaccumulation than particulate form in the estuarine snail *Peringia ulvae* [155], the freshwater snail *Lymnaea stagnalis*, the water flea *Daphnia magna* [156], and the freshwater oligochaete *Lumbriculus variegatus* [157].

Environmental dynamics such as dissolution stage or aggregation stage of the nanoparticles influence the uptake, bioaccumulation, and toxicity of the particles. For example, in aquatic snails, dissolved phase is responsible for the total uptake of silver, copper oxide, and zinc oxide nanoparticles [63, 156–158].

Croteau et al. have proved that aggregation can also affect bioavailability [63, 159] have measured the aggregation dependence of bioavailability of silver, copper oxide, and zinc oxide nanoparticles in the snail *L. stagnalis*. In mussels, aggregation was reported to increase the bioavailability [90].

When engineered nanomaterials enter into the environment, they are likely to mingle with the food or diet of animals and other organisms. These particles integrate with food material by aggregation and sorption processes. Hence, considering the dietary exposure of nanomaterials and its biological effects is equally important to assess ecological and human health risks. Croteau et al. revealed that isotopically labelled foodborne zinc oxide nanoparticles efficiently assimilated in the freshwater snails. Agglomeration does not interfere with the bioaccumulation and toxicity and resulted in lesser food consumption and impaired digestion. Consequently, developmental processes such as growth and reproduction will be affected resulting in population and community changes [159]. Additionally, Croteau et al. have reported the bioaccumulation and toxicity of copper oxide nanoparticles in freshwater invertebrate, *Lymnaea stagnalis*, following waterborne and foodborne exposure. It was concluded that diet-borne copper oxide nanoparticles are more deleterious readily than waterborne particles [63].

In *Daphnia magna*, single-walled carbon nanotubes and copper oxide nanoparticles accumulate in the gut as revealed using TEM imaging [59, 60]. Growth and reproductive ability of freshwater flea, *Daphnia magna* are affected due to titania and zinc oxide nanoparticles in a chronic study of 12 days [160]. Zhao et al. have done acute and chronic toxicity studies on the effects of waterborne and diet-borne silver nanoparticles and its bioaccumulation in a model freshwater cladoceran, *Daphnia magna*. A 48-hour acute study showed high bioaccumulation at 500 *μ*g/L. In a chronic study (21 days), waterborne silver nanoparticles significantly inhibited the growth. The chronic effects of silver nanoparticles might be due to the low food quality of algae contaminated with silver nanoparticles. This study has emphasised the significant of chronic toxicity studies in assessing the environmental risk of nanoparticles [161].

Oysters are an ecologically significant group of filter feeders of marine water. They can serve as a perfect toxicology model for illustrating the potential impacts of nanoparticles to marine organisms. *Crassostrea virginica* is an ideal marine organism for toxicity assessment of nanoparticles. Fullerene (concentration ≥100 ppb) was reported to impair embryonic development and cause lysosomal destabilisation associated with reproductive failure. Within 4 hour of exposure, fullerene particles concentrate on the lysosome-rich hepato-pancreatic tissues. Thus, endocytic and lysosomal pathways are the mechanisms by which fullerene exerts its toxic effects. It is also obvious that disturbance in the lysosomal pathway can cause chronic effects to the health and environment [162]. Mean chronic concentration that is hazardous to a given percentage of freshwater species (typically 95%) values were reported to be 0.2 mg/L for fullerene, 4.8 mg/L for CNTs, 1.2 *μ*g/L for silver nanoparticles, and 2 mg/L for titania nanoparticles [163].

Zerovalent nano-iron are capable of rapid dissolution in water such that the released iron particles exceed safe limits of NOECs established for dissolved Fe. This was proved in an acute study conducted using sperms of three key marine invertebrate species *Mytilus galloprovincialis, Ciona intestinalis*, and *Psammechinus milliaris*. In vitro fertilisation postexposure resulted in a decrease in success of fertilisation, delayed embryogenesis, and a disruption in the embryo development [164].

From the perspective of predator-prey interactions, a prey item with nanoparticles in the gut lumen will function as a nanomaterial-borne/contaminated food for the predator. In this context, the uptake, consequent assimilation, and the trophic transfer of dietary nano-CeO_2_ particles (containing gamma emitting radioisotope Cerium-141) along a freshwater food chain of alga, prawn, and snail were reported by Cresswell et al. [55]. The study asserted the rapid elimination of ceria nanoparticles in snail and the prawn and revealed the absence of assimilation in these organisms.

There are very few reports on ecotoxicology studies on environmentally relevant algae. Algae (*Desmodesmus subspicatus*) on exposure to titanium nanoparticles in growth inhibition test showed that the surface structure/matrix of plant cell walls could act as a surface to grow nanoparticles [165]. Nanoparticles show adsorption to the surfaces of aquatic sediments, algal mats, biofilms, soils, and even the exterior surfaces of organisms [166].

### 5.2. Aquatic Ecosystem-Vertebrates

Nanoparticle uptake in the fish gills is almost similar to that in the mucus layer and reported to occur primarily via vesicular endocytosis and less likely by diffusion and transporter-mediated processes. The probability of susceptibility of different organs to nanotoxicity are in the order gills > gut > liver > brain. Nanoparticles are excreted via hepato-biliary mechanism or kidney. But the glomerular excretion is not common for all fishes. The molecular weight cutoff for glomerular filtration is 60 kDa. Hence nanoparticles of few nanometres on par with 60 kDa will undergo glomerular filtration in most but not all the fish verities. Exceptionally, the glomerular kidneys of stenohaline marine and the sea water-adapted fish in the hyperosmotic environment cannot excrete the nanoparticles. The production of less urine or no urination is the reason for the hyperosmotic environmental species. However, the effect of nanomaterials on the fish varies depending on the fish habitats. For example, marine water shows high salinity or the ionic strength which cause aggregation. Even fishes dwelling in hardwater and benthic species at the sediment interface will be exposed to aggregates of nanoparticles rather than nanoparticulate suspension or dispersed nanoparticles. Soft water (freshwater) on the hand possesses nanoparticles that are stabilised by organic matter such as fulvic acid and humic acid [167]. Fish epithelial surface contains mucus which is analogous to the mucus of other vertebrates. The majority of the mucus layer (95%) is made of water, while mucoproteins (with highly conserved sialic acid, carboxylic acid, and sulphated residues) and electrolytes constitute the remaining proportion. Nanoparticles entangle strongly with mucoproteins, and the binding strength is more for nonspherical morphology. For example, single-walled carbon nanotubes were reported to bind strongly with the gill mucous of trout [93, 125]. From the mucous layer, the nanoparticles move across the epithelial layer of cells to the blood (transcellular movement) and then move across different cells via tight junctions (paracellular movement). Gut epithelia are capable of absorbing the nanoparticles through endocytosis. Albeit gills are the major portal entry, other routes are buccal cavity, olfactory openings, eyes, and urinary/genital openings. Nanoparticles' entry through these routes may damage nerve endings and cause damage to the retina [167].

Overall, the gills, gut, liver, and brain are the possible target organs for the toxic effects of some manufactured NPs in fish. The mechanism of toxicity includes oxidative stress, inflammation, tumor formation in the liver, disturbances in the ion homeostasis, and vascular injury [84]. For example, titania nanoparticles absorbed via gills induce oxidative stress and inflammation in the internal organs with a concomitant rise in the reactive oxygen species and inflammatory factors.

### 5.3. Effects of Soilborne Nanomaterials on Terrestrial Biota

Schultz et al. have demonstrated the trans-generational sensitivity in nematodes (*Caenorhabditis elegans*) exposed to silver nanoparticles for 10 generations. Epigenome was thought to be involved in the sensitivity transfer [168]. Carbon-based nanomaterials such as carbon nanotubes, fullerene, and graphene were reported to be nontoxic or less toxic to soil organisms such as earthworm and microbes [169–171]. Carbon nanotubes (double walled) impregnated into soil exerts toxicity to larva of amphibian. Similarly, the larvae of amphibian are prone to the toxicity of iron oxide, titania, zinc oxide, and copper oxide nanomaterials [172, 173]. Oxidised copper nanoparticles may proceed through food chains. For example, copper nanoparticles move from soil end enter into earthworm, eliciting toxic effects at a concentration >65 mg·Cu·kg^−1^ soil [174, 175].

### 5.4. Target Organs for Water and Diet-Borne Nanomaterials

Gomes et al. have revealed the bioaccumulation of copper oxide nanoparticles using the mussel *Mytilus galloprovincialis*. Digestive gland is the major site of bioaccumulation of copper oxide nanoparticles. Copper nanoparticles bioaccumulate and exert their toxicity by eliciting oxidative stress. This could be characterised by assaying lipid peroxidation, activities of antioxidant enzymes, and metallothionein levels. Copper nanoparticles are capable of lowering the activity of superoxide dismutase with a concomitant raise in lipid peroxidation and metallothionein content [176].

Nanoparticles manufactured for biomedical and industrial applications are usually functionalised to resist high ionic strength-mediated aggregation. Those particles exhibit high colloidal stability due which they show environmental persistence. As a result, these particles are expected to induce toxicity in aquatic system. The gut epithelium is the target for surface-stabilised metal nanoparticles. For example, *Corbicula fluminea*, a globally distributed clam, is known to uptake and accumulate gold nanoparticles functionalised with bovine serum albumin in the gut [56]. Silver nanoparticles functionalised with citrate molecules are predominant in estuarine sediments which are habitat and food for deposit feeders. *Nereis diversicolor* (deposit feeder) fed with citrate-capped silver nanoparticles were capable of accumulating the particles in their gut epithelium. The nanoparticles appear as electron-rich zones in the apical plasma membrane, endocytic pits, and in endosomes. These zones can be resolved using TEM [125]. Copper nanoparticles induce swelling of goblet cells, necrosis in the mucosa layer, and vacuole formation in the gut [177].

Nanomaterials are capable of eliciting immunotoxicity and neurotoxicity. In fishes, brain histochemistry gets altered due to nanoparticle toxicity in trouts. Copper nanoparticles elicit toxicity in the cell bodies of the neurons in telencephalon and alter the mesencephalon layer integrity, together with cerebral aneurysms [177]. Ramsden et al. have studied the sublethal effects of dietary exposure to titania nanoparticles in juvenile rainbow trout *Oncorhynchus mykiss*. Titania nanoparticles showed bioaccumulation and persistence in brain as evidenced by an inhibition in the activity of Na^+^K^+^ ATPase, alteration in Cu-Zn homeostasis, without affecting the growth and haematological parameters. In addition, gills and intestine showed enhanced lipid peroxidation [178].

The fact that the liver of aquatic organisms is also a target for nanoparticles was proved by Al-Bairuty et al. in trout models [177]. Hepatitis-like injury and cells with pyknotic nuclei are the toxicity indicators.

Nephrotoxicity of waterborne copper nanoparticles was also reported by Al-Bairuty et al. Trouts treated with copper nanoparticles shoed renal tubular epithelial injuries and altered Bowman's space in the kidney. Last but not the least, copper nanoparticle treatment in trout causes changes in the area of skeletal muscle fibers there by affecting muscular homeostasis [177]. Gills of the rainbow trout exhibits hyperplasia, aneurisms, and necrosis in the secondary lamellae [177].

Olfactory canals are also targets for nanoparticle-induced toxicity. In fishes, the accumulation of nanoparticles in olfactory canals impairs sensation pertaining to alarm chemicals. The antipredator behavioural responses of juvenile rainbow trout (*Oncorhynchus mykiss*) to trout alarm substance were investigated. The effect of nanoparticles includes a delay in freeze response and altered swimming activity. Change in behaviour was accompanied by a significant increase in the ratio of oxidised to reduced glutathione in the brains of fish, specifying some systemic oxidative stress. However, the morphology of olfactory bulb rosette was not affected [179].

External tissues of aquatic organisms are also targets for metal nanoparticles in water media! Sensory lateral line functions get altered in zebra fish (*Danio rerio*) due to the adverse effects of nanoparticles present in the water. The reason is probably the changes in the number of lateral lines neuromasts (LLNs) and rheotaxis behaviour. Copper nanoparticles reduced LLN. Copper nanoparticles and silver nanoparticles were capable of reducing LLN number and rheotaxis behaviour. This results in loss of sensory perception, resulting in altered foraging behaviours, increased susceptibility to predation, and avoidance of fish migrations [180]. This study is a good example for external tissue-mediated toxicity behaviour of metal nanoparticles in aquatic biological system.

### 5.5. Nano-Bio Interface

Knowledge on the reaction dynamics at the interface of nanomaterials with cells, subcellular organelles, and biomolecules is essential for understanding the toxic effects of nanomaterials. Cellular dynamics is also significant from the perspective of safe use of nanomaterials. Nanoparticles interact with subcellular organelles such as membrane, mitochondria, nucleus, lysosomes etc. Moreover, vital biomolecules such as DNA, proteins, and lipids are also sites for nanoparticle interaction which results in the formation of protein corona, particle wrapping, and free energy. Therefore, it is essential to ensure safe manufacture, usage, and disposal of nanomaterials in the marketplace.

Considering the wide target for nanomaterial interaction and interface formation, certain general mechanism of toxicity has been reported. Possible mechanism of the toxicity of nanomaterials on biological system are as follows:

- disruption of membrane structural integrity;
- interference with membrane potential;
- oxidation of proteins;
- genotoxicity;
- interruption of energy transduction;
- generation of reactive oxygen species and pro-oxidant status.

Nanomaterials are capable of generating reactive oxygen species that are involved in oxidising fatty acid chains of membranes by interacting with the double bonds. As a result, the integrity, the fluidity, and the membrane potential get altered [181].

Silver nanoparticles bind to biomembranes altering their permeability and potential. Silicon NPs and fullerene derivatives are also capable of inducing membrane damage altering the permeability and transport processes [182]. Silver nanoparticles and negatively charged nanomaterials were able to enter into lysosomes of the cells present in fish gills and intestinal lining by causing loss of membrane integrity, lysosomal damage, dysfunction, and autophagy [183, 184]. Silver nanoparticles interact with thiol groups of sulphur-containing amino acids in the vital enzymes and interact with DNA and prevent replication [185]. Silver nanoparticles are also capable of interacting with DNA and lipids causing their degradation [182]. Polyvinylpyrrolidone (PVP)-functionalised fullerene generates singlet oxygen that can cause lipid peroxidation and other cell damage [186].

Single-walled carbon nanotubes are known to block ion channels of the cell membrane [187]. Nanoparticles are capable of targeting gate keepers such as the epithelial barrier of the lungs, intestine, and the endothelial barrier of the blood vessels. For example, carbon nanotubes were reported to impair the function of biological barriers. Smaller sized particles follow paracellular route of transport while larger particles followed energy-dependent transcellular route of transport into the barrier cells [166, 188].

Iron-sulphur cluster are cofactors for many cellular enzymes. These clusters are targets for nanomaterials. Nanomaterials generate reactive oxygen species which impairs the function of the clusters. Further, the disulphide bridges are formed between the sulphur-containing amino acids of the enzymes leading to an impairment in the structure and the function of the enzymes [189].

Though nanomaterials such as quantum dots are used for DNA labelling and imaging, they induce nick in supercoiled DNA [190]. Quantum dots due to their small size pass through the nuclear pore complex targeting histone proteins that play an important function in cell cycle regulation and tumorigenesis [191]. Core-shell structures are capable of causing bioaccumulation and cause adverse effect due to biopersistence. Semiconductor quantum dots such as CdSe, CdTe, CdSeTe, ZnSe, InAs, or PbSe contain noble or transition metals in their core. Similarly, quantum dots such as CdS or ZnS contain metals in their shell [192, 193].

Fullerenes bind DNA and cause structural deformation, destabilisation, and functional impairment of the DNA molecules and cleavage [194–196]. Titanium dioxide nanoparticles (present in sunscreen lotion) generate oxygen radicals that can nick supercoiled DNA [197]. Tungsten carbide and silver nanoparticles induce genotoxicity (micronuclei formation) in mammalian cells. Mechanism of action includes oxidative stress and interference with microtubules and actin filaments during cell division [198–200].

Iron oxide nanoparticles establish steric interactions with the cytoskeleton network and interfere with the polymerisation and maturation of actin fibers, thereby inhibiting the cell differentiation and migration [201]. Tungsten nanofibers and zinc oxide nanoparticles enter into the epithelial lining of the hepatopancreas and frog embryo enterocytes causing oxidative stress and alteration in the structure and function of the cell junctions [202, 203].

Engineered nanoparticles such as titania, silver, polystyrene, and carbon nanoparticles were reported to cause mitochondrial dysfunction thereby impairing energy production [204]. Electron transport chain, oxidative phosphorylation, and energy transduction are vital processes of the cell. Nanoparticles interfere with these processes indirectly or directly. Indirect process involves binding of nanomaterials to membrane and subsequent alteration in membrane integrity. Direct process involves redox-sensitive nanoparticle that binds to membrane-bound electron carriers and pulls out electrons from the transport chain. Fullerene and cerium dioxide nanoparticles are capable of interfering with the cellular energy transduction [205–207].

As mitochondria plays a role in regulating apoptosis (programmed cell death), nanomaterials are capable of impairing the regulatory of mitochondria. Quantum dots and silica nanoparticles induce developmental malformation in the zebra fish embryo heart. Gold nanoparticles induce malpigmentation in the eyes of zebrafish leading to altered swimming behaviour. Both these effects were reported to be due to interference with the apoptosis signalling [208–210].

Considering the toxicological effects of several nanoparticles, several *in vitro* and *in vivo* experimental studies have been done to identify the potential compounds which could combat the toxicity of specific nanoparticles. For example, *in vivo* studies have proved the efficacy of nanoparticles of bisdemethoxycurcumin analog in ameliorating MWCNT-induced toxicity [211]. It has been reported that fenugreek extract and quercetin combat petrol exhaust nanoparticle-induced lipid peroxidation and oxidative stress in red blood cells [212]. Cardioprotective effect of quercetin was reported in petrol exhaust nanoparticle-induced toxicity *in vitro* [213].

### 5.6. Phytotoxicity of Nanoparticles

Wang et al. have demonstrated the trans-generational effects of ceria nanoparticles using tomato plants. Tomato plants were treated with low concentrations of CeO_2_ (10 mg·L^−1^) and the seeds from the generation plant were collected and used to grow second-generation seedlings. The second-generation plants were relatively smaller and weaker, as indicated by their smaller biomass, lower water transpiration, and slightly higher reactive oxygen species content together with higher accumulation of ceria [214]. Similarly, ceria nanoparticles are toxic to wheat as indicated by morphological and biochemical effects, reductions in chlorophyll, delayed flowering, and increased catalase and superoxide dismutase activities [215]. Soilborne ceria nanoparticles show bioaccumulation in the roots and root nodules of soybeans. Ceria also shows bioaccumulation in the roots and shoots of corn plants [216, 217]. Ceria nanoparticles induces alteration in nutrient assimilation in corn and bioaccumulation in soybean [218, 219].

Titania, silver, and zinc oxide nanoparticles were added to soil samples. The amended soil was used as media for the legume *Medicago truncatula*. These nanoparticles were reported to reduce the root nodulation in legume and also altered the microbial community in the soil [218]. Soil under field conditions spiked with titania and zinc oxide nanoparticles bind into the cells of wheat plants. Titania nanoparticles bind strongly to the cell wall of wheat plant cells and decreased the biomass. Zinc oxide nanoparticles that are absorbed not only decreased the biomass but also decreased the activities of soil enzymes protease, catalase, and peroxidase showing the adverse effect on soil quality [219].

Engineered iron oxide nanoparticles were absorbed and accumulated by pumpkin (*Cucurbita maxima*) plants [220]. Arbuscular mycorrhizal fungi (AMF) establish a mutualistic symbiosis with majority of the terrestrial plants. Iron oxide nanoparticles significantly reduced mycorrhizal clover biomass by reducing the glomalin content and root nutrient acquisition of AMF [221]. In plants, nanoscale aluminium was reported to induce phytotoxicity by suppressing rhizogenesis probably through high solubility [222].

## 6. Nanomaterials as Vectors for Other Contaminants

Several contaminants such as radioactive elements, polychlorinated compounds [223], potentially toxic elements (PTE) [224], and pesticides [225] present in the sediments or suspended as solids in water undergo sorption on nanoparticle's surface through physical sorption (which involves van der Waals interaction), electrostatic interaction, ion-exchange, chemical adsorption (involves bond formation) etc. The sorption process of various contaminants may passivate the nanoparticle's active surfaces affecting environmental behaviour and toxicity of not only of the nanoparticle but also the adsorbed contaminants by influencing their dissolution and solubility kinetics [226]. Nanoparticles act as carriers of contaminants and enter in the organism as a particle-contaminant complex. Thus, the complexed contaminants are released inside the organisms, thereby increasing its bioavailability and toxicity by the “Trojan horse effect.”

Recent studies have reported the following:

1. Adsorption of polybrominated diphenyl ethers on titanium dioxide and zinc oxide nanoparticles through aromatic ether groups and Br suppresses the agglomeration of nanoparticles in natural water resulting in enhanced transport and exposure of pollutants to aquatic organisms [227, 228].
2. Sorption of certain antibiotics like levofloxacin and ciprofloxacin on graphene oxide (GO) enhances the mobility and transport of these antibiotics through porous media which may increase their risks to ecological receptors and could also cause groundwater contamination [229].
3. The pluronic acid-modified single-walled carbon nanotubes (PA-SWCNTs) act as a carrier in the porous media and facilitate the transport of gold nanoparticles [230].
4. Similarly, the adsorption of polycyclic aromatic hydrocarbons, PAHs (naphthalene, phenanthrene), and aldrin through electrostatic attraction and surface complexation process on TiO_2_ and MWCNTs surface increases the aqueous phase concentration of these hydrophobic organic pollutants as compared to the “real” partitioning due to the octanol-water partitioning [231].
5. The hydrophobic dissolved organic matter (DOM) coating on Ag-Ag_2_S and CeO_2_ nanoparticles reduced the adsorption capacity of methylene blue by around 54% and 70%, respectively. The blockage of nanoparticle surface active sites with DOM reduces the adsorption of dye [232].
6. The adsorption of organochlorines (atrazine, hexachlorobenzene, pentachlorobenzene, and 3, 3′, 4, 4′-tetrachlorobiphenyl) by TiO_2_ nanoparticles increases the bioaccumulation of these contaminants to algae [223].
7. The co-exposure of nanoparticles (such as TiO_2_, Ag, Al_2_O_3_, graphene, and CNTs) with PAHs, organochlorine pesticides (OCPs), and polybrominated diphenyl ether (PBDE) in soil to *Ipomoea* aquatic, *Cucumis sativus* L., *Zea mays* L., *Spinacia oleracea* L., and *Cucurbita moschata* promotes the uptake and accumulation of organic contaminants in crop plants [233].
8. Co-exposure of graphene nanoparticles at 50 mg/kg level (4–20 nm·size) substantially increased the bioaccumulation of organic contaminants through adsorption, followed by co-transfer into crop tissues [233].
9. Pulmonary surfactant (PS) altered the air-liquid interfacial properties of carbon nanoparticles which may increase the pulmonary risk of atmospheric exposure of both PAHs and carbon nanoparticles [234].
10. Co-exposure of ZnO Nanoparticles and Pb^2+^ enhanced the Pb accumulation in all major organs of mice, induced excessive production of hepatic ROS and pro-inflammatory cytokines, and aggravated liver injury [235].

Apart from the above, there is an emerging concern for microplastics in the aquatic ecosystems, which upon interaction with nanoparticles can either passivate or accelerate the environmental hazards. The interaction of microplastics with nanoparticles can modify the properties such as size, surface chemistry, stability, conductivity, solubility, persistence resulting fate, transport, and toxicity of both nanoparticles and microplastics [236]. Polystyrene (PS) microplastics can effectively remove the Ag nanoparticles in the aquatic environment by monolayer adsorption through electrostatic interaction [237]. The co-presence of TiO_2_ nanoparticles in polystyrene microplastic suspensions decreases microplastic transport and promotes their rapid deposition in quartz sand by the formation of heteroagglomerates [238]. It has been reported that the co-exposure of PS and Ag nanoparticles to *Chlamydomonas reinhardtii* and *Ochromonas danica* stimulated the toxicity of pollutants to freshwater algae through synergistic interactions [239]. Similarly, the chronic exposure of MP and Au nanoparticle mixture to planktonic crustacean *Daphnia magna* hinders development, reproduction, and eventually leads to death.

Thus, it could be concluded that the adsorption of contaminants on the surface of the nanoparticles not only modifies the environmental fate of both the contaminant and nanoparticles but also alters the ecotoxicity of nanoparticle-contaminant complexes.

## 7. Trophic Transfer of Nanoparticles

The biomagnification of gold nanomaterials in a simulated tobacco (*Nicotiana tabacum*)-tobacco hornworm (*Manduca sexta*) caterpillar food chain [240] has been reported. This biomagnification raises concerns regarding the potential for humans to be exposed to nanomaterials via trophic transfer.

This work was followed by other studies that reported trophic transfer of nanomaterials in other simulated food chains including:

1. Earthworm (*Eisenia fetida*) to Bullfrog (*Rana catesbeiana*) [241].
2. Zucchini (*Cucurbita pepo*) to Cricket (*Acheta domesticus*) [242].
3. Lettuce (*Lactuca sativa*) to Cricket to Darkling beetles (*Tenebrionoidea*) [243].

In spite of the fact that each of the aforementioned studies reported trophic transfer, the concentration of nanomaterials transferred were small and the biomagnification reported in the tomato-hornworm study was not observed. However, recently, the biomagnification of nanomaterials was again reported in a terrestrial food chain, with CeO_2_ nanomaterials accumulated in kidney bean (*Phaseolus vulgaris*), plants biomagnifying in Mexican bean beetles (*Epilachnavarivestis*), as well as in consumers of the beetles, spined soldier bugs (*Podisusmaculiventris*) [244]. Altogether, these studies indicate that trophic transfer of nanomaterials occur at least in some small amount in most terrestrial food chains, with certain terrestrial organisms and food chains being particularly susceptible to biomagnification, although the reasons that some organisms are more likely to biomagnify nanomaterials remain unclear.

## 8. Conclusion

There are only limited knowledge and limited review papers focusing on the environmental hazards and exposure of nanomaterials, which in turn creates large uncertainties in understanding the risk. This type of review will result in the database showing the risk of eco-nanotoxicity, the opportunities and challenges in the determination and the prevention of eco-nanotoxicity. The degrees of uncertainties in the data can be analysed by using this type of review. Regulatory agencies can avail this type of review to rightly classify the nanoparticles and to manage nanomaterials as compared to their bulk counterparts. Hence, our review systematically focused on the source of exposure, environmental and biological dynamics, and the adverse effects of nanoparticles whose production rate is constantly in hike. This approach will reveal many research targets for nanotechnology community and will be a frontline to address environmental issues. This review will afford a reference for future studies and guide researchers for structuring objectives to tackle the nanotoxicology-related issues and to reduce further emissions. We infer that this review will direct the scientists and researchers towards a new era of green nanotechnology.

## 9. Future Perspectives

Suitable analytical metrology for detecting the physiochemical properties and the quanta of transformed nanoparticles in the environmental matrices is needed. This can to a certain extent be achieved by integrating and customising the currently available sophisticated techniques. Also, suitable methodology to isolate and quantify the bioavailable proportions of nanoparticles is essential for determining the toxicity in aquatic and terrestrial organisms. As the marketing of nanoparticle-based products are in hike, strict testing and regulation should be enforced to regulate the production, handling, and disposal of nanoparticles. As the research on nanobiotechnology is increasing, the animal experimentation pertaining to biomedical applications of nanomaterials should be properly regulated. More focused research and experiments can be done on the teratogenic effects of different types of nanoparticles. Environmental-friendly protocols can be followed during the synthesis, applications, and the disposal of wastewater and devices fabricated with nanoparticles.

## Figures and Tables

**Figure 1:** Sourced of nanoparticles and their environmental entry.

**Table 1:** Techniques used for the characterisation of nanomaterials in environmental samples.

S. no	Techniques	Applications in environmental nanotoxicology assessment
1	Dynamic light scattering	Gives an idea of the particle sizes in the whole dispersion
2	Differential centrifugal sedimentation	To generate fractions containing different particle sizes
3	Size exclusion chromatography	Chromatographic fractions are generated according to molecular weight, enabling plots of size distribution
4	Field flow fractionation technique	High-resolution particle size distributions and separation of subfractions
5	Electrophoretic mobility	To determine the surface properties of nanoparticles that is net surface charge
6	N_2_ absorption (BET analysis)	For measuring the specific surface area of particles
7	Gravimetry	To filter the environmental samples
8	Turbidimetry	Particle concentration can be estimated

**Table 2:** Biological effects of various nanoparticles on aquatic organisms.

S. no.	Nanoparticles	Biological effects
1	Silver nanoparticles	Alters membrane permeability and potential. Interacts with thiol groups of sulphur-containing amino acids in the vital enzymes, interact with DNA and prevent replication.
2	Silicon NPs and fullerene derivatives	Induces membrane damage altering the permeability and transport processes. Negatively charged nanomaterials, lysosomal damage, dysfunction, and autophagy.
3	Polyvinylpyrrolidone (PVP)-functionalised fullerene	Generates singlet oxygen that can cause lipid peroxidation and other cell damage.
4	Single-walled carbon nanotubes	Blocks ion channels of the cell membrane.
5	Carbon nanotubes	Targets the gate keepers such as the epithelial barrier of lungs, intestine, and the endothelial barrier of the blood vessels.
6	Quantum dots	Targets the nuclear pore complex and histone proteins and impairs cell cycle regulation.
7	Core-shell structures	Induces bioaccumulation and bio persistence (CdSe, CdTe, CdSeTe, ZnSe, InAs, PbSe, CdS, ZnS).
8	Fullerenes	Causes structural deformation, destabilisation, and functional impairment of the DNA molecules.
9	Titanium dioxide nanoparticles (present in sunscreen lotion)	Generates oxygen radicals that can nick supercoiled DNA.
10	Tungsten carbide and silver nanoparticles	Induces genotoxicity.
11	Iron oxide nanoparticles	Interferes with the polymerisation and maturation of actin fibers. Inhibits the cell differentiation and migration.
12	Tungsten nanofibers and zinc oxide	Alters the structure and function of the cell junctions in fish embryo
13	Fullerene and cerium dioxide	Interferes with the cellular energy transduction
14	Quantum dots and silica nanoparticles	Induces developmental malformation in the zebra fish embryo heart.
15	Gold nanoparticles	Induces malpigmentation in the eyes of zebrafish leading to altered swimming behaviour.

## Data Availability

The datasets used and/or investigated during the current study are available from the corresponding authors upon reasonable request.
